The article "Analyzing Neck Circumference as a Tool for Evaluating Overweight and Obesity in Chinese Adolescents" was retracted in 2023. Reasons: unreliable results or conclusions; concerns about the data; concerns about the peer review; concerns about the citations.

# Analyzing Neck Circumference as a Tool for Evaluating Overweight and Obesity in Chinese Adolescents

**DOI:** 10.1155/2021/1274627

**Published:** 2021-10-06

**Authors:** Hui Wang

**Affiliations:** Department of Physical Education, Xiamen University TKK College, Zhangzhou 363105, China

## Abstract

Overweight and obesity at an early age are important criteria for predicting chronic diseases. Each anthropometric method available to assess obesity has its limitations. Recently, neck circumference (NC) has received greater attention as a new evaluation index. This study aimed to investigate the relationship between NC and overweight in Chinese Yi adolescents. A total of 647 Chinese Yi male and female students, aged 13–18 years, were randomly selected from a junior high school and a senior middle school in Leshan, Sichuan Province of China. The measurement indexes included height, weight, waist circumference (WC), and NC, and clinical information was collected by trained physicians. The neck cutoff values were determined through the receiver operating characteristic (ROC) curve and the area under the curve (AUC). The correlation among NC, body mass index (BMI), and WC was determined by Pearson's correlation coefficient. The ROC analysis revealed that the AUC values were 0.79–0.95 for boys and 0.83–0.91 for girls. The correlation among NC, BMI, and WC in obese boys and girls was higher than 0.70 in both genders. In addition, the NC cutoff values of high BMI ranged from 31.0 cm to 36.1 cm for boys and 31.2 cm to 34.5 cm for girls, respectively. There was a significant positive correlation between NC and obesity in Chinese Yi adolescents. The NC can be used as an additional index to predict the obesity of Chinese Yi adolescents.

## 1. Introduction

Overweight and obesity can lead to a variety of chronic diseases, such as metabolic syndrome, hypertension, and diabetes mellitus. Obesity also increases the incidence of cardiovascular diseases and cancer and reduces physical fitness. In children, the incidence of obesity has increased up to 300% over the last 30 years. The National Health and Nutrition Examination Survey (2009–2010) found 30% of children between 5 and 19 years of age to be overweight. Obesity varied from 15 to 40% in different European populations [1, 2].

Obesity has grown rapidly in Chinese children and adolescents in the past 30 years. The rate of overweight and obesity among Chinese children and adolescents within 6–17 years of age was 9.6% and 6.2%, respectively, in 2012, and this was increased by 113.3% and 195.2%, respectively, in 2002 [3]. Likewise, the abdominal obesity rate was 12.29% in Chinese minority groups. Several studies have investigated the association between obesity and its markers with a variety of chronic diseases and even correlation with malignancies that may threaten public health in China. From 1985 to 2015, for 7–18-year-old Chinese Yi individuals (formerly called Lolo or Wuman) living in Leshan, Sichuan Province of China, the obesity rate of males increased from 0.08% to 2.65%, while the obesity rate of females increased from 0.10% to 2.02%, respectively [4, 5]. An important approach to control obesity and overweight would be to develop a practical method of diagnosis for this disease which is simple, reliable, and low cost for the assessment of adolescents, especially in primary healthcare. There are several anthropometric methods used to assess obesity and overweight. ome techniques are applicable for evaluation of obesity like measurement of waist, hip circumference, weight, and height; however, there is still controversy about the effectiveness of some methods for measuring overweight and obesity in children and adolescents [6–8].

Body mass index (BMI, weight/height^2^) is considered to be the main anthropometric measure for evaluating overweight due to its low cost and ease of application. However, despite these advantages, several studies have shown numerous shortcomings about its application to the correct diagnosis of obesity composition and that the BMI cannot clearly distinguish the distribution of body fat [9, 10]. One major shortcoming is that BMI indexes both fat mass (FM) and fat-free mass (FFM) and, within populations, the ratio of FM to FFM varies considerably at any given BMI. At the same time, BMI cannot reliably index regional body composition, and it is understood that centrally deposited and visceral FM contributes significantly to variability in metabolic risk [11]. The use of imaging methods (e.g., MRI and X-ray) to measure adipose tissue depots is the best way but may be limited by cost, time, and access to equipment. Body composition proxies that go beyond BMI, but are simple, scalable, and reliably indicative of relative disease risk, have thus been sought [12, 13]. Several studies have revealed that waist circumference (WC), waist-to-hip ratio (WHR), and waist-to-height ratio (WHtR) are suitable indicators to evaluate chronic metabolic diseases associated with obesity and overweight [10]. In addition, neck circumference (NC) is a new indicator to assess obesity in children, when compared with WC, WHR, and WHtR. It mainly reflects the upper body subcutaneous fat (UBSF) distribution to estimate central obesity, and results have revealed that the method is easy to accomplish, convenient, and accurate [14]. NC has also received wide interest as a proxy for upper body FM depots, with studies conducted in children, adolescents, and adults in a range of populations. Across these studies, NC correlated with other anthropometric parameters (e.g., WC and BMI), as well as single and clustered cardiometabolic risk factors, and performed well as a tool to identify those with, or at risk of, metabolic syndrome [15–17].

There are 55 minorities in China. However, few studies have focused on the correlation between NC and obesity, especially for the Yi nationality. The Yi nationality is the sixth-largest minority in China, with a population of 8,714,393 (2010 National census statistics). The region of Liangshan Yi Autonomous Prefecture is the main stronghold of Chinese Yi individuals. In the context of the rapid pace of population movement in modern society, the pace of population integration has further accelerated. Maintaining the uniqueness of the physical characteristics of ethnic minorities has become very urgent [18, 19]. Therefore, investigating the unique characteristics of minorities is necessary. However, to the best of our knowledge, no study has investigated the reference data on NC in adolescents of Chinese Yi. Therefore, the present study aimed to investigate the correlation among NC, WC, and BMI in Chinese Yi adolescents and determined the best NC cutoff points to identify obesity in Chinese Yi adolescents, thereby improving the Chinese national physical health database.

The rest of the paper is organized as follows: Section 2 describes the methodology of the proposed work, Section 3 illustrates the results, the results are discussed in Section 4, and finally, the conclusion is given in Section 5.

## 2. Materials and Methods

### 2.1. Subject

This study was approved by the Research Ethics Committee of the Xiamen University, Zhengzhou, China. In the present study, a total of 647 Chinese Yi adolescents, who were 13–18 years old, were recruited. Among these subjects, 305 subjects were girls and 342 subjects were boys, and these children were admitted to a middle school and a primary school in Leshan. The participants have no other disorders, and children with trauma, thyroid disease, superficial lymph node enlargement of the neck, and cervical malformations that can affect the normal development of the neck were excluded from the present study.

### 2.2. Anthropometric Measurements

Anthropometric measurements are quantitative measurements of the muscle, bone, and adipose tissue used to evaluate the structure of the body. The core elements of anthropometry are height, weight, body mass index (BMI), and body circumferences such as waist, hip, and limb. In this study, the anthropometric measurements, including height, weight, WC, and NC, were obtained. These subjects were instructed to wear light clothing and no shoes. The height and weight tests were performed under the “National student physical health survey report 2010” [20] physique and health test conditions, and BMI was calculated by dividing weight (kg) by height (cm) squared (m^2^). During the WC test, the subjects were instructed to stand upright with their arms open and sagging, to reveal their abdominal skin. The WC test point was 2 cm above the navel, the position of the body side was located between the lower ribs and the top of the iliac crest, and the measured value was recorded up to 0.1 cm. Data were collected using a weighing machine, height measuring scale, and flexible measuring tape. Height was measured with help of a stadiometer, and each individual was trained to stand barefoot and head held in horizontal plane to the nearest 0.1 cm. The weight of each subject was measured by using a calibrated electronic weighing scale, to the nearest 0.1 kg. Neck circumference was measured between the mid-cervical spine and mid-anterior neck, using a flexible measuring tape with the subjects in the standing position, head held erect, and eyes facing forwards and neck in the horizontal plane at the level of the most prominent position, the thyroid cartilage. Informed consent was obtained from the head of the school and assent was obtained from the school students. Informed consent was also taken from parents. Approval was obtained from the Institutional Ethics Committee before instating the study. The demographic and anthropometric data are represented in Table 1.

### 2.3. Statistical Analysis

The ROC analysis was used to determine the predictive validity of NC and evaluate the cutoff values for identifying overweight or obese children. The ROC curve represents a plot of the true-positive rate (sensitivity) against the false-positive rate (specificity) [21, 22]. The AUC describes the probability that a test would correctly identify a pair of patients. Normally, the AUC is less than 0.5, indicating that the method or index is almost inefficient. When the AUC is closer to 1, this means a better diagnosis [23]. According to the Youden Index, if sensitivity and specificity are diagnostically equally significant, the Youden index will specify the performance at a given cutoff. The Youden index is a common summary measure of the ROC curve. The maximum value of the Youden index is 1 (perfect test), and the minimum is 0 when the test has no diagnostic value. Pearson's correlation coefficient was used to determine the relationship among BMI, WC, and NC. Obesity was distinguished according to the “Overweight and obesity screening criteria for Chinese school-aged children and adolescents” [24–27]. The descriptive statistics were produced by both of the genders for age, weight, height, BMI, NC, and WC. Continuous variables were represented as mean ± standard deviation. The *T*-test was used to compare the mean anthropometric values between boys and girls. The results were considered statistically significant when *p* < 0.05. All the statistical analyses were carried out using Statistical Package for Social Sciences Software (SPSS, Windows version 20.0, Chicago, IL, USA).

## 3. Results

The present study recruited 647 participants between 13 and 18 years. Among the 647 subjects, 342 were male subjects, the mean age observed was 14.38 years, and 305 were females. The results of the descriptive statistics (Table 1) revealed that the age between boys and girls has no significant difference (*p* > 0.05). The weight, height, NC, and WC were higher in boys than in girls, but the BMI was lower in girls. All anthropometric values were significantly different in both genders (*p* < 0.05).

Table 2 shows Pearson's correlation coefficients between NC and the other anthropometric values, including age, weight, height, BMI, and WC. Overall, the NC of obese boys and girls and other body measurement correlation coefficients were higher than those in the normal group. The correlation coefficient of NC and age in normal boys and girls was 0.204 (r = 0.204) and 0.275 (r = 0.275), respectively, which shows a weak relationship. However, there is no significant difference in both genders (*p* > 0.05). Likewise, the correlation coefficient of age and obese boys and girls was 0.213 (r = 0.213) and 0.360 (r = 0.360), respectively. However, the correlation between NC and height in the normal group and obese group had no significant difference (*p* > 0.05), and the maximum correlation coefficient was only 0.246, presenting a low correlation between these groups. In the obese group, NC revealed a moderate or high correlation (Min = 0.71, Max = 0.84) with weight, BMI, and WC in both genders. The correlation coefficient for the obesity group was higher than that for the normal group, showing an obvious difference (*p* < 0.001).

Tables 3 and 4 represent the results of the ROC analysis in obese boys and girls for NC, respectively. These results show that the AUC values of boys ranged from 0.79 to 0.95, while the values for girls ranged from 0.83 to 0.91 (Table 4). Furthermore, the AUC values were close to 1 in both gender and all ages. The cutoff values of the NC of obese boys ranged from 31.0 cm to 36.1 cm, while the cutoff values of the NC of obese girls ranged from 31.2 cm to 34.5 cm, respectively. The sensitivity interval of obese boys was 70.0%–87.5%, and the specificity interval was 74.8%–87.3%. Likewise, the sensitivity interval of obese girls was 80.3%–88.6%, and specificity was 72.1%–87.5%, respectively. These results reveal a significant difference in both genders (*p* < 0.01).

The correlation coefficient among BMI, WC, and NC is shown in Table 5. It was found that the correlation coefficients among BMI and NC (BMI-NC) ranged from 0.76 to 0.88 for boys and 0.81 to 0.91 for girls, respectively. Similarly, the correlation coefficient of NC and WC varied from 0.74 to 0.85 for boys and ranged from 0.75 to 0.90 for girls. Likewise, the correlation coefficients between BMI and WC ranged from 0.69 to 0.87 for boys and 0.71 to 0.83 for girls, respectively. All correlation coefficients have a significant difference in both gender and age (*p* < 0.001). In genral, NC showed a strong relationship with BMI and WC in both males and females.

## 4. Discussion

At the beginning of the 20^th^ century, overweight and obesity were rare. In the year 1997, the World Health Organization (WHO) officially reported obesity as a global epidemic. According to the WHO report, 65% of the world's population live in countries where overweight and obesity kill more people than underweight. The incidence of obesity is rising at an alarming speed, and the harmful effects are prominent [5–7]. Obesity has become the major problem that affects global public health, and pose a greater threat to the health of young people. The WHR is commonly used to recognize individuals with obesity and overweight. However, the WC is less specific and can vary in the postprandial period, in the menstrual period, and according to bowel function. NC reflects the deposits of adipose tissue in the neck and can be used as the best indicator of subcutaneous adipose tissue in the upper body [11, 12]. Previous studies have suggested that abdominal adiposity among children and adolescents has an increasing trend in developing or developed countries [15]. At present, there are many indicators to evaluate obesity. In 1957, the wideness of the neck was used to evaluate the distribution of upper body fat for the first time, and the distribution of neck fat was revealed to be closely correlated to whole body fat [17]. Later, NC became a prominent research hotspot for researchers. The neck is the junction between the trunk and head not covered by clothing and is convenient for measurement. In addition, NC measurements are less invasive than the measurement of WC and less cumbersome than assessing BMI.

In the present study, a significant association between NC and other anthropometric values of obesity was found in both gender and all ages. These results also show that the NC measurement can be used as an easy and convenient method for overweight and obesity surveys on the Chinese Yi nationality. Many researchers have found that the advantages of NC mainly focus on the following three points when compared with other methods. First, WHtR and WC methods may be time consuming and culturally or environmentally problematic, especially in the winter season, because clothes have to be removed for obtaining accurate and precise measurements [16]. Second, NC is not affected by other physical indicators. For example, previous studies have suggested that BMI cannot accurately identify the specific distribution of fat because it is affected by height, age, and race differences [18]. In the present study, it was found that the correlation coefficient of NC and height was lower than 0.30, demonstrating that height has little effect on NC. Third, NC can effectively identify recessive obesity. Recessive obesity refers to the normal look from the physical form, whereas fat mainly accumulates in the visceral part [19]. Even if WC is normal, the visceral fat may be excessive because fatness is implicated, and the measurement of WHR has the same limitations [19].

The present study revealed that the AUC values for boys ranged from 0.85 to 0.94, while the AUC values for girls ranged from 0.83 to 0.91, respectively, and the minimum value of the AUC was 0.83, which was close to 1. This means that NC performed better in diagnosing obesity. It was also reported that there was a higher correlation between NC and BMI and WC (*r* > 0.70). These results were consistent with a previous study, in which the increase in obesity in the adolescent group was positively correlated with the increase in NC [20]. This suggests that NC is a simple and convenient measurement to identify children and adolescents who are overweight and obese [21]. Other studies have also suggested that NC can be used with great reliability to predict overweight and obese children and identify those with a high BMI [22]. In general, the comprehensive results of this study confirmed that there is a significant correlation between NC and obesity in children and adolescents. Based on the present results (Tables 4 and 5), the cutoff values for NC in boys ranged from 31.0 cm to 36.1 cm, and these could be regarded as obese groups, while the cutoff values for NC in girls ranged from 31.2 cm to 34.5 cm, and these could be considered as obese groups. The NC cutoff values in the present study were lower in boys who were 13–18 years old when compared with Han adolescents and other country-related data [23]. The reason may be due to ethnic differences and socioeconomic factors. Generally, the measurement of NC was more easy, convenient, and accurate, when compared with other measurements, in terms of evaluating overweight and obesity in adolescents. In addition, NC had a significant correlation with obesity in adolescents. Therefore, NC could be regarded as an optimal index to predicted obesity in Chinese Yi adolescents. The limitation of the present study was that the present subjects were recruited from the city of Leshan, and the inclusion date for children living in rural areas may have affected these results. This was the first attempt that examined the value of NC in a wide range in Chinese Yi children for both genders, and these results can improve the Chinese national physical health database.

## 5. Conclusion

Overweight and obesity can lead to a variety of chronic diseases, such as metabolic syndrome, cardiovascular disorders, hypertension, and diabetes mellitus. The present anthropometric methods for the evaluation of obesity have their limitations. In this study, the relationship between NC and overweight was investigated in Chinese Yi adolescents. A total of 647 Chinese Yi male and female students, aged 13–18 years, from a junior high school and a senior middle school in Leshan, Sichuan Province of China, participated in this study. The measurement indexes included height, weight, WC, BMI, and NC. The correlation among NC, body mass index (BMI), and WC was determined by Pearson's correlation analysis. The present study validated that NC is a simple and easy tool to screen and identify overweight and obese adolescents when compared to other methods used for obesity determination. Results revealed a significant positive correlation among NC, WC, and BMI in excess weight among Chinese Yi adolescents. The NC could be used as an additional index for evaluating overweight and obesity in Chinese Yi adolescents. The present study concluded that NC is a valuable tool for screening obesity among adolescents with reasonable sensitivity and specificity.

## Figures and Tables

**Table 1:** General characteristics of the study population.

Variable	Boys	Girls	*p*
Age (years)	15.4 ± 1.6	15.5 ± 1.5	0.517
Weight (kg)	47.2 ± 10.8	46.6 ± 11.0	0.001
Height (cm)	158.4 ± 11.3	152.8 ± 11.2	0.001
BMI (kg/m^2^)	18.7 ± 5.1	19.9 ± 4.8	0.002
NC (cm)	32.9 ± 3.0	31.5 ± 3.2	0.014
WC (cm)	67.4 ± 10.7	64.5 ± 11.2	0.001

BMI: body mass index; NC: neck circumference; WC: waist circumference. *T*-test was used to compare the difference between boys and girls. *p* values <0.05 were considered significant.

**Table 2:** The relationship between NC and other anthropometric variables in normal and obese adolescents by gender.

Variable	Normal boys		Obese boys		Normal girls		Obese girls	
	*r*	*p*	*r*	*p*	*r*	*p*	*r*	*p*
Age	0.204	0.043	0.213	0.060	0.275	0.035	0.360	0.440
Height (cm)	0.183	0.106	0.430	0.074	0.246	0.080	0.160	0.133
Weight (kg)	0.569	0.001	0.745	0.001	0.651	0.001	0.805	0.001
BMI (kg/m^2^)	0.588	0.050	0.726	0.001	0.783	0.001	0.710	0.001
WC (cm)	0.541	0.001	0.769	0.001	0.675	0.001	0.840	0.001

**Table 3:** AUCs, optimal cutoff values, sensitivities, and specificities for NC associated with obesity in 13–18-year-old boys.

Age (years)	*N*	AUC (95% CI)	Cutoff	Sensitivity (%)	Specificity (%)	*p*
13	57	0.95 (0.87–0.98)	31.0	72.2	80.1	0.008
14	57	0.90 (0.74–0.92)	33.3	70.0	76.0	0.001
15	58	0.94 (0.79–0.98)	33.7	71.4	85.3	0.001
16	56	0.79 (0.68–0.89)	34.9	72.7	87.3	0.001
17	57	0.92 (0.82–0.99)	35.2	87.5	83.0	0.001
18	57	0.89 (0.84–0.99)	36.1	86.3	74.8	0.001

**Table 4:** AUCs, optimal cutoff values, sensitivities, and specificities for NC associated with obesity in 13–18-year-old girls.

Age (years)	*N*	AUC (95% CI)	Cutoff	Sensitivity (%)	Specificity (%)	*p*
13	52	0.91 (0.77–0.98)	31.2	86.6	75.0	0.005
14	51	0.83 (0.69–0.98)	32.0	71.1	87.5	0.003
15	51	0.84 (0.73–0.95)	32.5	76.6	74.9	0.003
16	51	0.86 (0.51–0.99)	33.7	80.3	76.7	0.001
17	50	0.90 (0.81–0.99)	33.1	85.7	72.1	0.001
18	50	0.87 (0.68–0.91)	34.5	88.6	78.4	0.001

**Table 5:** Pearson's correlation coefficients of anthropometric indexes by age and gender.

	BMI-NC			NC-WC			BMI-WC		
Age	Male	Female	*p*	Male	Female	*p*	Male	Female	*p*
13	0.84	0.81	<0.001	0.74	0.79	<0.001	0.87	0.78	<0.001
14	0.80	0.88	<0.001	0.82	0.90	<0.001	0.75	0.80	<0.001
15	0.83	0.85	<0.001	0.76	0.83	<0.001	0.78	0.83	<0.001
16	0.82	0.91	<0.001	0.85	0.75	<0.001	0.69	0.77	<0.001
17	0.76	0.83	<0.001	0.77	0.84	<0.001	0.84	0.71	<0.001
18	0.88	0.81	<0.001	0.82	0.79	<0.001	0.74	0.82	<0.001

## Data Availability

The data used to support the findings of this study are included within the article.
